# Ectopic Expression of a Maize Hybrid Down-Regulated Gene *ZmARF25* Decreases Organ Size by Affecting Cellular Proliferation in *Arabidopsis*

**DOI:** 10.1371/journal.pone.0094830

**Published:** 2014-04-22

**Authors:** Chuan Li, Cheng Wang, Lingxue Meng, Jiewen Xing, Tianya Wang, Hua Yang, Yingyin Yao, Huiru Peng, Zhaorong Hu, Qixin Sun, Zhongfu Ni

**Affiliations:** 1 State Key Laboratory for Agrobiotechnology and Key Laboratory of Crop Heterosis and Utilization (MOE), Beijing Key Laboratory of Crop Genetic Improvement, China Agricultural University, Beijing, China; 2 National Plant Gene Research Centre (Beijing), Beijing, China; Department of Agriculture and Food Western Australia, Australia

## Abstract

Heterosis is associated with differential gene expression between hybrids and their parental lines, and the genes involved in cell proliferation played important roles. *AtARF2* is a general cell proliferation repressor in *Arabidopsis*. In our previous study, two homologues (*ZmARF10 and ZmARF25*) of *AtARF2* were identified in maize, but their relationship with heterosis was not elucidated. Here, the expression patterns of *ZmARF10 and ZmARF25* in seedling leaves of maize hybrids and their parental lines were analyzed. The results of qRT-PCR exhibited that *ZmARF25* was down-regulated in leaf basal region of hybrids. Moreover, overexpression of *ZmARF25* led to reduced organ size in *Arabidopsis*, which was mainly due to the decrease in cell number, not cell size. In addition, the cell proliferation related genes *AtANT, AtGIF1* and *AtGRF5* were down-regulated in 35S::*ZmARF25* transgenic lines. Collectively, we proposed that the down-regulation of *ZmARF25* in maize hybrid may accelerate cell proliferation and promote leaf development, which, in turn, contributes to the observed leaf size heterosis in maize.

## Introduction

Heterosis is defined as advantageous quantitative and qualitative traits of offspring over their parents, and the utilization of heterosis principles has been a major practice for increasing productivity of plants and animals [1]. In spite of its importance and successful application, the underlying molecular mechanism for heterosis is still needs to be elucidated [2]–[5]. Studies on plant form evolution suggest that phenotype evolution often proceeds through changes in the spatial and temporal patterns of gene expression [6]. Theoretically, all the genes in hybrid are inherited from its two parental lines, but hybrid performance or phenotype can be quite different from its parents, thereby, demonstrating heterosis [7], [8]. Therefore, the alteration of gene expression in hybrids may be responsible for hybrid vigor [4], [8]. Up to date, genome wide gene expression profiles of different organs or tissues between hybrids and their parents in plants have been analyzed [9]–[15], and all possible modes of gene action were observed, including additivity, high- and low-parent dominance, underdominance, and overdominance [9]–[15]. To gain further insight into the possible roles of differentially expressed genes between hybrid and its parental lines in plant development and heterosis, the functions of some differentially expressed genes have been characterized, and some of which may contribute to the observed heterosis. For example, overexpression of wheat hybrid up-regulated gene (*ADP-ribosylation factor*, *TaARF*) in *Arabidopsis* displayed increased growth rates during the seedling and adult stages [16]. Overexpression of Larix hybrid up-regulated gene *LaAP2L1*, a member of the AP2/EREBP transcription factor family, led to markedly enlarged organs and heterosis-like traits in *Arabidopsis* [17]. Expression of an up-regulated protein ZmACT2 in dry embryos of maize hybrid in *Arabidopsis* partially complemented the low germination phenotype in the *Atact7* mutant [18].

Heterosis affects nearly any trait in nearly every hybrid, hence one of the major challenges for expression analysis is deciding which tissue to be analyzed [19], [20]. It was proposed that seedling leaves can be used as a model system to investigate the molecular basis of maize heterosis, because it is commonly observed that hybrids produce larger leaf areas than their corresponding parental lines [20]–[24]. At the cellular level, a crucial effect of leaf size heterosis is manifested by primarily increases in cell number, not cell size [25]–[27]. Recent study provided molecular evidence for the relationship between cell proliferation and heterotic maize growth. For example, the expression level of maize *CNR* gene, ortholog of *fruit weight 2.2* (*fw2.2*) in tomato, was founded to be negatively correlated with growth activity and hybrid vigor [28]. Collectively, it reveals that the study of cell number control is eminently important to understanding the underlying mechanism for leaf size heterosis.

In *Arabidopsis*, auxin signaling plays a vital role in leaf growth and development processes and some key genes, including *AtARF2*, *AtARF7 and AtARF19*, have been identified [29]–[31]. In our previous study, 31 maize genes that encode ARFs (Auxin Response Factors) were identified in maize genome, and phylogenetic analysis demonstrated that two of them, *ZmARF10* and *ZmARF25*, were homologous to *Arabidopsis* growth repressor *AtARF2* [32]. In this study, the expression patterns of *ZmARF10* and *ZmARF25* in seedling leaves of maize hybrids and their parental lines were investigated and the function of hybrid down-regulated gene *ZmARF25* was characterized. Our data showed that ectopic expression of *ZmARF25* in *Arabidopsis* led to reduced organ size, indicating that the alteration of auxin signaling pathway might play an important role in maize leaf size heterosis.

## Materials and Methods

### Plant Materials and Growth Conditions

Maize inbred lines Mo17, B73, Zong3, 87-1 and their hybrids Mo17/B73, B73/Mo17, Zong3/87-1, 87-1/Zong3, B73/Zong3, Zong3/B73, B73/87-1 and 87-1/B73 were used for this study. Maize seeds were imbibed at 28°C in the dark, and the seeds after germination were selected with the same length of coleoptile (2.0 cm) to grow in hydroponic culture on a 16 h light/8 h dark cycle, at a temperature of 29°C and 25°C for the light and dark cycle, respectively. In maize leaf, the mature zone is composed of fully differentiated cells and cell division is restricted to the growing zone composed of immature cells [19], [33]. Therefore, thirty millimeters from the base of the third leaves and twenty millimeters from the tip of the same leaf of a seedling 5 days after germination (DAG) were dissected and harvested for RNA extractions.

*Arabidopsis* (Col-0) seeds were sterilized by a 60 s 70% ethanol treatment followed by 1% NaClO within 10 min, four washes in distilled water, and chilled at 4°C for 3 days. Seeds were sown on half-strength Murashige and Skoog (MS) plates with 3% sucrose and 0.8% agar in a culture room at 22°C under a 16/8 light/dark cycle. After germination, 10-day-old *Arabidopsis* seedlings were transplanted and grown at a density of four plants per pot containing a mixture of soil and vermiculite (2∶1) at 22°C under a 16/8 light/dark cycle with 70% relative humidity.

### Leaf Area Measurements

Leaves were scanned using ImageScanner (GE Healthcare, USA), and measured with a public domain image analysis software (ImageJ version 1.32; http://rsb.info.nih.gov/ij/). For maize leaf area measurements, the third leaves were harvested in the morning (10∶00–10∶30 am) and experiments were done in three biological replicates and 10 plants of each genotype were analyzed for each replicate. The *t*-test was used to determine the significance of the differences in leaf areas between hybrid and the corresponding mid-parental value. The mid-parent heterosis (MPH) was calculated using the following formula: MPH = (F_1_−mid-parental value)/mid-parental value in %, where F_1_ is the average value of hybrid, and the mid-parental value is the average value of the two parents.

Ten 30-day-old *Arabidopsis* plants of each transgenic line and wild-type were selected randomly for the fully expanded fifth leaf area measurements. The *t*-test was used to determine the significance of the differences in leaf area between transgenic plants and wild-type plants.

### Histological Analysis

After the area measurements, the fully expanded fifth leaves of the ten 30-day-old *Arabidopsis* plants of each transgenic line and wild-type were used for epidermal cell size measurements. Leaves were first boiled in water for 10 min to kill the cells, and then immersed in 95% ethyl alcohol, after decolorized, they were transferred to hot (96°C) 85% lactic acid for 8 min. Finally, the leaves were transferred to room temperature lactic acid and examined using a Nikon Stereo Microscope. The number of epidermal cells was determined in an area of 0.58 mm^2^ in the middle region of the fifth leaf blade. The average cell size was measured by dividing 0.58 mm^2^ by the number of epidermal. The total number of cells per leaf was calculated by dividing the leaf area by the average cell size. Statistical calculations were performed with Microsoft EXCEL.

### Isolation of DNA and Total RNA

Total DNA was extracted by the cetyltrimethylammonium bromide (CTAB) method [34] with minor modifications. Total RNA was extracted using a standard Trizol RNA isolation protocol (Invitrogen, USA), and then treated with RNase-free DNaseI (Promega, USA) to remove genomic DNA. The amount and quality of the total RNA were verified by electrophoresis on a 1% agarose gel. The concentration of RNA was measured using a NanoDrop spectrophotometer (ND- 1000; NanoDrop Technologies). First-strand cDNA synthesis was performed using 2 µg of DNase digested total RNA with oligodT15 primer according to the manufacturer’s protocol for RT-PCR first-strand synthesis (TaKaRa, Japan).

### Quantitative RT-PCR Analysis

Quantitative RT-PCR (qRT-PCR) using SYBR Green PCR master mix (TaKaRa, Japan) was performed using CFX96 Real-Time PCR Detection System (Bio-Rad Laboratories, Inc., USA). Specific primers for qRT-PCR analysis were listed in Table S1. The PCR efficiency of all primer pairs was determined from standard curve experiments. PCR conditions consisted of an initial step at 95°C for 3 min followed by 40 cycles of 95°C for 15 s, followed by 60°C for 15 s, and then 72°C for 30 s. For amplification product specificity, a melting curve was generated at the end of each run, and verified by agarose gel electrophoresis of PCR products. All reactions were run in triplicate, and each reaction was completed with a melting curve and amplification curve analysis to confirm the amplification specificity. Ct values were determined using the CFX96 software with default settings. Differences between the Ct values of target gene and *Actin* were calculated as ΔCt = Ct_target gene_−Ct*_Actin_*, and the relative expression levels of target genes were determined as 2^−ΔCt^. For each sample, PCR was performed on three biological replicates. The average values of 2^−ΔCt^ were used to determine difference in gene expression. *Actin* was amplified as an endogenous control. Statistical analysis of the difference in the relative expression levels of target genes was performed by using *t*-test.

### Gene Cloning and Sequence Analysis

PCR was performed using the ZmARF25-F/R primer pair from the first-strand cDNA from the B73 seedling leaves. PCR conditions consisted of an initial step at 94°C for 5 min followed by 35 cycles of 94°C for 25 s, 58°C for 25 s, and 72°C for 2 m 45 s; and then a final step at 72°C for 10 min. The PCR products were confirmed by visualization of the samples by electrophoresis on 1% agarose gel and stained by Ethidium bromide. The samples were extracted with MinElute Gel Extraction Kit (Qiagen, Germany), and these purified PCR products were cloned into pGEM-T plasmid vector (Promega, USA). Three clones were subsequently sequenced (Invitrogen, USA). The online tools, Open Reading Frame Finder (http://www.ncbi.nlm.nih.gov/gorf/gorf.html), Compute pI/Mw (http://web.expasy.org/compute_pi/), and InterPro (http://www.ebi.ac.uk/interpro/), were used to analyze the nucleotide and amino acid sequences.

### Vector Construction and Plant Transformation

The coding region of *ZmARF25* was introduced into pDONR221 vector using Gateway BP clonase enzymemix (Invitrogen, USA) with the following primer pair: Gate-25-F and Gate-25-R (Table S1). To construct overexpression vector 35S::*ZmARF25*, the fragments were transferred from the pDONR221 vectors to pB2GW7 vector by Gateway LR recombination (Invitrogen, USA). This construct was transformed into *Arabidopsis* (Col-0) via the floral dip method using Agrobacterium tumefaciens strain GV3101 [35]. Transgenic plants were selected on 1/2 MS medium containing herbicides (Basta). The herbicide resistant seedlings were transferred to a mixture of soil and vermiculite (2∶1) and generated homozygous lines by self-fertilization. Statistical analysis of the difference in traits between transgenic plants and wild-type plants was performed by using *t*-test.

## Results

### Comparison of Maize Leaf Area between Hybrids and their Parental Lines

Previous studies revealed that maize hybrid exhibited heterosis in leaf size [24]. In this study, dynamic growth patterns of maize hybrid Mo17/B73 and its inbred parental lines were investigated in terms of the third leaf area and mid-parent heterosis (MPH) was calculated. The results exhibited that leaf areas of hybrid Mo17/B73 were significantly larger than its parental lines at 8, 10 and 12 DAG. Remarkably, MPH (72.00%) at 8 DAG was much higher than that of 10 and 12 DAG (60.50% and 58.26%) [Figure S1]. Thus, the third leaf areas of eight hybrids and their parental lines at 8 DAG were further measured and compared. It can be seen that the leaf areas of all hybrids were significantly larger than those of their parental lines at 8 DAG [Figure 1A].

**Figure 1:** The third leaf areas and expression patterns of *ZmARF10* and *ZmARF25* between maize hybrids and their parental lines . (A) The third leaf area and mid-parent heterosis at the 8 DAG. H represents mid-parent heterosis (MPH). **refers to significant at *p*<0.01, data are represented as the mean ± SE (n = 3). (B–D) Expression patterns of *ZmARF10* and *ZmARF25* in different leaf regions of maize hybrids and their parental lines at the 5 DAG. B, C and D indicated as basal region, tip region and basal region, respectively. *β-actin* was used as an endogenous control. Data are represented as the mean ± SE (n = 3), *refers to significant at *p*<0.05, **refers to significant at *p*<0.01.

### Identification of a Hybrid Down-regulated Gene *ZmARF25* in Maize Seedling Leaves

To gain insight into the relationship of *ZmARF10* and *ZmARF25* with leaf size heterosis, expression patterns of these two genes in the third leaves of hybrids Mo17/B73 and B73/Mo17 and their parental lines. Considering of the time lag between differential gene expression and the observed heterosis of leaf size at 8 DAG, the third leaves at 5 DAG were selected for qRT-PCR analysis. As shown in Figure 1B, the relative expression levels of *ZmARF25* in the basal region of Mo17/B73 and B73/Mo17 hybrids were significantly lower than the levels observed in parental lines, whereas no significant differences in the expression patterns of *ZmARF10* were observed in these hybrids. Most notably, no obvious expression alterations were detected for *ZmARF10* and *ZmARF25* in the leaf tip regions of the hybrids and their parental lines [Figure 1C]. Furthermore, the expression patterns of *ZmARF25* between other hybrids and their parental lines were also investigated and we observed that *ZmARF25* was down-regulated in the leaf basal regions of Zong3/87-1, 87-1/Zong3, B73/87-1, 87-1/B73 and Zong3/B73, but not B73/Zong3 [Figure 1D]. Therefore, *ZmARF25* was selected for further investigation.

To obtain the cDNA with complete open reading frame (ORF) corresponding to *ZmARF25*, cDNAs from B73 seedling leaves were amplified with ZmARF25-F/R primer pair and one unique PCR fragment of about 2500 bp was produced (data not shown). The PCR products were cloned into pGEM-T and three clones were sequenced. One 2552 bp fragment was obtained and no nucleotide polymorphisms were detected for all sequenced clones. Sequence analysis revealed that the PCR product contains a complete ORF, which encodes a polypeptide of 801 amino acids with a calculated molecular mass of 89.79 kD and isoelectric point of 6.09, which was consistent with our previous study [32]. Structure analysis exhibited that ZmARF25 has a typical ARF-type structure with a conserved DNA-binding domain (DBD) that consists of a plant-specific B3-type subdomain and an ARF subdomain required for efficient *in vitro* binding to the auxin response elements (AuxREs) in the N-terminus, a typical carboxy-terminal dimerization domain (CTD) with both III and IV subdomains and a middle region (MR) that might function as a repression domain (RD) since it is enriched in serine (S) [Figure 2] [36]–[39].

**Figure 2:** Amino acid sequences alignment and graphical representation for domain organization of ZmARF25 proteins. Identical amino acids are indicated by asterisks, amino acid position numbers are indicated on the right. B3 domain is marked with green box, ARF subdomain is marked with blue box, MR is marked with red box, and subdomain III and IV are marked with purple box and orange box, respectively.

### Functional Analysis of *ZmARF25* in *Arabidopsis*

To investigate the possible function of *ZmARF25*, overexpression *Arabidopsis* transgenic plants were generated and herbicide-resistant T_0_ transformants were transferred into soil and grown in a greenhouse to obtain segregating T_1_ progeny for genetic analysis. Of the 21 transformants, eight overexpression lines showed a 3∶1 segregation pattern for herbicide resistance, among which four (35S::*ZmARF25* #1–4) were selected for further analysis. As shown in Figure 3A, the insertion of the overexpression vector was confirmed by genomic PCR. *ZmARF25* is a homologue of *AtARF2* in *Arabidopsis* [32], the relative expression levels of exogenous gene *ZmARF25* and endogenous gene *AtARF2* in the transgenic and wild-type plants were analyzed by qRT-PCR. The results showed that different expression levels of *ZmARF25* were observed in these overexpression lines, but the transcription of *AtARF2* in the transgenic lines was not affected [Figure 3B]. Subsequent analysis was conducted using these T_3_ homozygous transgenic plants. As shown in Figure 4, 35S*::ZmARF25* #1–4 transgenic lines displayed markedly decreased leaf areas, shorter siliques and plant height with smaller inflorescences and flowers in comparison with wild-type. Further analysis revealed that the size of the fifth leaves of 35S::*ZmARF25* plants was decreased by approximately 60∼80% as compared to wild-type [Figure 4D]. In addition, the plant height and the silique length of transgenic plants were about 40–60% and 56% of that of wild-type, respectively [Figure 4E, F]. Collectively, these data indicated that overexpression of *ZmARF25* in *Arabidopsis* decreased the size of aerial organs by inhibiting organ growth and development.

**Figure 3:** Overexpression of *ZmARF25* in *Arabidopsis*. (A) The genomic PCR results for four homozygous T_3_ transgenic plants (35S::*ZmARF25* #1–4) using *Bar* gene specific primer. PCR products were determined visually by running on 1% agarose gel and stained by Ethidium bromide. Col represents wild-type and #1–4 represent 35S::*ZmARF25* transgenic lines, which is the same in Figure 3B; “+” represents the recombinant plasmid. (B) Relative expression levels of *ZmARF25* gene in four homozygous T_3_ transgenic lines. Total RNA was isolated from the 30-day-old aerial of *Arabidopsis*. Data are represented as the mean ± SE (n = 3). *ACTIN2* was used as an endogenous control.

**Figure 4:** Morphology of 35S::*ZmARF25* and wild-type plants. Morphology of (A) leaf size, (B) Inflorescences, flowers and siliques and (C) plant height. Statistics of (D) fully expended fifth leaves area, (E) siliques and (F) plant height. Col represents the wild-type; #1–4 represent the four 35S::*ZmARF25* transgenic lines; data are represented as the mean ± SE (n = 10). *t*-test compared with the wild-type control: **refers to significant at *p*<0.01.

To determine whether it is cell number or cell size, or both that contribute to the changed leaf size in transgenic lines, we observed and compared the size and number of cells in the fully expended fifth leaves between 35S::*ZmARF25* and wild-type plants. The results showed that there was no distinct difference in cell size between the *ZmARF25* overexpression and wild-type plants [Figure 5A, B], whereas cell number of 35S::*ZmARF25* plants was significantly lower when compared to wild-type plants [Figure 5C], indicating that the decrease in cell numbers, not cell size, was associated with the diminution of leaf size in 35S::*ZmARF25* plants.

**Figure 5:** Histological analysis of fully expanded fifth leaves of 35S::*ZmARF25* and wild-type plants. (A) Epidermal cells of the fully expanded fifth leaves of *35S::ZmARF25* and wild-type plants. The statistics of (B) epidermal cells size and (C) cell number per leaf. Fully expanded fifth leaves of wild-type transgenic plants were analyzed. Data are represented as the mean ± SE (n = 10). *t*-test compared with the wild-type control: **refers to significant at *p*<0.01.

### Expression Analysis of Organ Size-associated Genes between 35S::*ZmARF25* Transgenic Lines and Wild-type

To elucidate the underlying regulation mechanism of *ZmARF25*, expression patterns of organ size-associated genes *AtANT*, *AtGIF1*, *AtGRF5* and *AtEXP10* between 35S::*ZmARF25* and wild-type plants were analyzed by qRT-PCR. The results showed that the expression levels of *AtANT*, *AtGIF1* and *AtGRF5* were significantly decreased in 35S::*ZmARF25* plants, whereas no obvious alteration of *AtEXP10* expression was observed [Figure 6]. In *Arabidopsis*, *AtANT*, *AtGIF1* and *AtGRF5* were reported to be involved in cell proliferation while *AtEXP10* played important roles in cellular expansion [40]–[44]. Collectively, it could be concluded that overexpression of *ZmARF25* inhibited the transcription of cell proliferation associated genes, which is consistent with the decreased cell numbers observed in 35S::*ZmARF25* plants.

**Figure 6:** Expression patterns of organ size related genes in 35S:*:ZmARF25* and wild-type plants. The aerial portions of 15-day-old seedlings were used for qRT-PCR analysis. *ACTIN 2* was used as the endogenous control. Col represents the wild-type; #1–4 represents the four 35S::*ZmARF25* transgenic lines. Data are represented as the mean ± SE (n = 3). *t*-test compared with the wild-type control: *refers to significant at *p*<0.05, **refers to significant at *p*<0.01.

## Discussion

### *ZmARF25* Repressed Organ Size by Decreasing Cell Numbers in *Arabidopsis*

Auxin response factors (ARFs) are transcription factors that bind with specificity to TGTCTC-containing AuxREs found in promoters of primary/early auxin response genes and mediate responses to the plant hormone auxin [36]–[39]. Genome-wide analysis revealed that *ARF* genes are represented by a large multigene family in plants [32], [45]–[49]. Most ARFs contain a conserved N-terminal DBD, a variable MR and a typical CTD [36], [37], [45]–[49]. The DBD specifically binds to the conserved AuXRE, the CTD is modular with amino acid sequence related to domains III and IV in Aux/IAA proteins, making it function as a dimerization domain among the ARFs or with several Aux/IAA proteins. The structure of MR determines whether the ARF acts as an activator or repressor. Activation domain (AD) of ARFs is usually enriched in glutamine (Q), serine (S) and leucine (L), while repression domain (RD) is enriched in either S, L and proline (P); S, L and/or glycine (G) or S [32], [39]. In this study, one hybrid down-regulated gene *ZmARF25* that encoded a typical ARF-type protein was identified in maize. Most notably, ZmARF25 has a MR enriched in S, indicating that it might act as a repressor. Our previous study indicated that ZmARF25 was homologous to AtARF2 in *Arabidopsis* and OsARF4 in rice [32]. *AtARF2* has been identified as a general repressor of cell division, one aspect of many biological processes regulated by auxin [29]. However, our knowledge about the functions and regulations of *ZmARF25* gene is quite limited. Here, we demonstrated that overexpression of *ZmARF25* in *Arabidopsis* resulted in significant size reduction of plant organs. Although the results of *ZmARF25* overexpression in *Arabidopsis* may not fully reflect its precise functions in maize, it is reasonable to assume that *ZmARF25* may be involved in maize growth and development process, which deserves for further investigation.

At the cellular level, organ size is determined by two developmental forces,cell proliferation and cell expansion, which partially overlap in time and are assumed to be coordinated [50]. Nevertheless, larger organ tends to be composed of more cells rather than bigger cells in different species [51]. In present study, we noted that overexpression of *ZmARF25* in *Arabidopsis* significantly decreased the cell number, resulting in smaller organs in 35S*::ZmARF25* transgenic plants when compared to wild-type. Recently, some regulatory genes that affect leaf development have been identified and characterized at the molecular level. For example, loss of *AtANT* function reduces the size of all lateral shoot organs by decreasing cell number [41]. *AtGIF* and *AtGRF5* act together and are required for the development of appropriate leaf size and shape by promoting and/or maintaining of cell proliferation activity in leaf primordial [42], [43]. On the other hand, expansins are thought to function in the control of plant cell growth, and leaf size was substantially reduced in antisense lines with suppressed *AtEXP10* expression, whereas overexpression of *AtEXP10* resulted in plants with somewhat larger leaves [44]. Remarkably, overexpression of *ZmARF25* repressed the expression levels of *AtANT*, *AtGRF5* and *AtGIF1*, whereas no significant alteration in *AtEXP10* expression was detected. Collectively, we speculate that *ZmARF25* regulates the process of cell proliferation by altering the expression of *AtANT*, *AtGRF5* and *AtGIF1* in *Arabidopsis*.

### Expression Patterns of *ZmARF25* in Maize Hybrids and their Parental Lines was Tissue and Genotype Dependent

Leaf differentiation proceeds basipetally (from tip to base) in a highly regular and continuous manner [52]–[54]. Maize leaves have a basal growing region, which is composed of immature cells, enclosed by older leaves [19], [33], [55]. Dynamics of the third leaf of maize seedling transcriptome and proteome along the maize leaf developmental gradient have been discussed. The results showed that genes and proteins expressed at the highest levels near the base of the leaf involved in cell wall biosynthesis, DNA synthesis, cell cycle regulation and chromatin structure regulation, protein metabolism, potential signaling proteins, auxin and brassinosteroid biosynthesis and signaling, respiratory pathways and vesicle transport [19], [56]. Interestingly, relative expression level of *ZmARF25* gene in the basal region of hybrids Mo17/B73 and B73/Mo17 was significantly lower than that of two parental lines. On the other hand, no significant alteration in expression was observed in the tip region, which is consistent with the observation that different regions within a leaf displayed different expression patterns [19], [56]. Taken together, we proposed that leaf basal region was the appropriate tissue for further investigation of the molecular basis of leaf size heterosis.

Recently, many studies have analyzed heterosis-associated gene expression in leaves of maize, rice and wheat [7]–[14], [20], but there has been no obvious consensus about genes that are differentially expressed in hybrids, which might be the result of significant differences in species, different genotypes within species, distinct tissues, experimental designs and statistical procedures applied [7]–[14], [20]. In this study, we noted that the *ZmARF25* gene was down-regulated in B73/Mo17, Mo17/B73, Zong3/87-1, 87-1/Zong3, B73/87-1, 87-1/B73 and Zong3/B73, but no significant expression difference was detected between B73/Zong3 and its parental lines, which may be attributed to the influence of maternal affect, because the mid-parent heterosis of hybrid B73/Zong3 was lower than that of Zong3/B73.

### Down-regulation of *ZmARF25* in Hybrids may Contribute to the Observed Heterosis for Leaf Size

Enlarged organ size, such as the increased leaf area, is an important feature of heterosis and also has a close relationship with the crop yield [12, 28 and 57]. A key observation made in maize heterosis was that the greater plant size is primarily (90%) due to increases in cell number, not cell size [25]. Recently study reported that transgenic over-expression of *Zea mays ARGOS1 (ZAR1)* enhanced maize organ growth [58]. The expression level of *CNR* gene was found to be negatively correlated with tissue growth activity and hybrid vigor [28], [57]. In this study, the expression patterns of *ZmARF10* and *ZmARF25* in maize hybrids and their parental lines were analyzed. We found that *ZmARF25* gene was down-regulated in hybrids. Moreover, 35S::*ZmARF25* transgenic *Arabidopsis* plants displayed markedly decreased aerial organ size in comparison with wild-type. Considering the decreased cell number in 35S::*ZmARF25* plant leaves, we proposed that the down-regulation of *ZmARF25* gene in maize hybrid could accelerate cell proliferation and promote leaf development, which, in turn, contributes to the observed heterosis for leaf size.

## Supporting Information

Figure S1 **The third leaf area of hybrid Mo17/B73 and its parental lines at 8 DAG, 10 DAG and 12 DAG.** H represents mid-parent heterosis (MPH). **refers to significant at *p*<0.01, data are represented as the mean ± SE (n = 3).
(TIF)

Table S1 **Gene specific primer pairs used in this study.**
(DOC)

## References

[1] BudakH (2002) Understanding of Heterosis. KSU J Science and Engineering 5(2): 69–75.

[2] LippmanZB, ZamirD (2007) Heterosis: revisiting the magic. Trends Genet 23: 60–66.1718839810.1016/j.tig.2006.12.006

[3] BirchlerJA, AugerDL, RiddleNC (2003) In search of the molecular basis of heterosis. Plant Cell 15: 2236–2239.1452324510.1105/tpc.151030PMC540269

[4] ChenZJ (2010) Molecular mechanisms of polyploidy and hybrid vigor. Trends Plant Sci 15: 57–71.2008043210.1016/j.tplants.2009.12.003PMC2821985

[5] BirchlerJA, YaoH, ChudalayandiS, VaimanD, VeitiaRA (2010) Heterosis. Plant Cell 22: 2105–2112.2062214610.1105/tpc.110.076133PMC2929104

[6] DoebleyJ, LukensL (1998) Transcriptional regulators and the evolution of plant form. Plant Cell 10: 1075–1082.966812810.1105/tpc.10.7.1075PMC1464652

[7] RomagnoliS, MaddaloniM, LiviniC, MottoM (1990) Relationship between gene expression and hybrid vigor in primary root tips of young maize (*Zea mays* L.) plantlets. Theor Appl Genet 80(6): 769–775.2422110710.1007/BF00224190

[8] SunQX, WuLM, NiZF, MengFR, WangZK, et al (2004) Differential gene expression patterns in leaves between hybrids and their parental inbreds are correlated with heterosis in a wheat diallel cross. Plant Sci 166: 651–657.

[9] HuangY, ZhangL, ZhangJ, YuanDJ, XuCG, et al (2006) Heterosis and polymorphisms of gene expression in an elite rice hybrid as revealed by a micriarry analysis of 9198 unique ESTs. Plant Mol Biol 62(4–5): 579–591.1694122110.1007/s11103-006-9040-z

[10] WeiG, TaoY, LiuGZ, Chen C LuoRY, et al (2009) A transcriptomic analysis of superhybrid rice LYP9 and its parents. Proc Natl Acad Sci U S A 106(19): 7695–7701.1937237110.1073/pnas.0902340106PMC2683082

[11] ZhangYH, NiZF, Yao YY Zhao J SunQX, et al (2006) Analysis of genome-wide gene expression in root of wheat hybrid and its parents using Barley1 Gene Chip. Progre Nat Sci 16(7): 712–720.

[12] Swanson-WagnerRA, JiaY, DeCook, BorsukLA, NettletonD, et al (2006) All possible modes of gene action are observed in a global comparision of gene expression in a maize F1 hybrid and its inbred parents. Proc Natl Acad Sci U S A 103(18): 6805–6810.1664110310.1073/pnas.0510430103PMC1447595

[13] PascholdA, JiaY, MarconC, LundS, LarsonNB, et al (2012) Hochholdinger F. Complementation contributes to transcriptome complexity in maize (*Zea mays* L.) hybrids relative to their inbred parents. Genome Res 22(12): 2445–2454.2308628610.1101/gr.138461.112PMC3514674

[14] PascholdA, MarconC, HoeckerN, HochholdingerF (2010) Molecular dissection of heterosis manifestation during early maize root development. Theor Appl Genet 120(2): 383–388.1952620510.1007/s00122-009-1082-6

[15] LiA, FangMD, SongWQ, ChenCB, QiLW, et al (2012) Gene expression profiles of two intraspecific Larix lines and their reciprocal hybrids. Mol Biol Rep 39(4): 3773–3784.2175091510.1007/s11033-011-1154-y

[16] YaoYY, NiZF, DuJK, Han ZF ChenY, et al (2009) Ectopic overexpression of wheat adenosine diphosphate- ribosylation, TaARF, increases growth rate in *Arabidopsis* . J Integr Plant Biol 51(1): 35–44.1916649210.1111/j.1744-7909.2008.00792.x

[17] LiA, ZhouY, JinC, SongWQ, ChenCB, et al (2013) LaAP2L1, a heterosis-associated AP2/EREBP transcription factor of Larix, increases organ size and final biomass by affecting cell proliferation in *Arabidopsis* . Plant Cell Physiol 54(11): 1822–1836.2400933510.1093/pcp/pct124

[18] GuoBJ, ChenYH, ZhangGP, XingJW, HuZR, et al (2013) Comparative proteomic analysis of embryos between a maize hybrid and its parental lines during early stages of seed germination. PLoS One 11 8(6): e65867 doi:10.1371/journal.pone.0065867 10.1371/journal.pone.0065867PMC367916823776561

[19] LiPH, PonnalaL, NeeruG, WangL, SiYQ, et al (2010) The developmental dynamics of the maize leaf transcriptome. Nature genetic 42(12): 1060–1067.10.1038/ng.70321037569

[20] Flint-GarciaSA, BucklerES, TiffinP, ErsozE, SpringerNM (2009) Heterosis Is Prevalent for Multiple Traits in Diverse Maize Germplasm. PLoS ONE 4(10): e7433 doi:10.1371/journal.pone.0007433 1982359110.1371/journal.pone.0007433PMC2757727

[21] SandeepKT, ReddyDM, SaidaNV, NagarajuC (2012) Heterosis for leaf, tassel characters and yield in single cross hybrids of maize (*Zea mays* L.). Journal of Progressive Agriculture 3(1): 152–154.

[22] JohnsonGR (1973) Diallel analysis of leaf area heterosis and relationships to yield in maize. Crop Sci. 13: 178–180.

[23] SpringerNM, StuparRM (2007) Allelic variation and heterosis in maize: how do two halves make more than a whole? Genome Res 17(3): 264–275.1725555310.1101/gr.5347007

[24] UchimiyaH, TakahashiN (1973) Kinetics of heterosis in growth of the leaf blade in *Zea mays* L. *Ann.* Bot. 37: 247–252.

[25] PavLrKovAE, RoorSB (1987) Cellular basis of heterosis for leaf area in maize. Can. J. Plant Sci. 67: 99–104.

[26] EastEM (1936) Heterosis. Genetics 21: 375–397.1724680110.1093/genetics/21.4.375PMC1208682

[27] Kiesselbach TA (1922) Corn investigations, in: Bulletin of the Agricultural Experiment Station of Nebraska, The University of Nebraska, Lincoln, Nebraska, U.S.A. 96–102.

[28] GuoM, RupeMA, DieterJA, Zou JJ SpielbauerD, et al (2010) Cell Number Regulator1 affects plant and organ size in maize: implications for crop yield enhancement and heterosis. Plant Cell 22(4): 1057–1073.2040067810.1105/tpc.109.073676PMC2879740

[29] SchruffMC, SpielmanM, TiwariS, AdamsS, FenbyN, et al (2005) The AUXIN RESPONSE FACTOR 2 gene of *Arabidopsis* links auxin signaling, cell division, and the size of seeds and other organs. Development 133: 251–261.1633918710.1242/dev.02194

[30] WilmothJC, WangS, TiwariSB, JoshiAD, HagenG, et al (2005) NPH4/ARF7 and ARF19 promote leaf expansion and auxin-induced lateral root formation. Plant J 43(1): 118–130.1596062110.1111/j.1365-313X.2005.02432.x

[31] KrizekBA (2009) Making bigger plants: key regulators of final organ size. Curr Opin Plant Biol 12(1): 17–22.1895183610.1016/j.pbi.2008.09.006

[32] XingHY, PudakeRN, GuoGG, XingGF, HuZR, et al (2011) Genome-wide identification and expression profiling of auxin response factor (ARF) gene family in maize. BMC Genomics 12: 178.2147376810.1186/1471-2164-12-178PMC3082248

[33] PalmerSJ, DaviesWJ (1996) An analysis of relative elemental growth rate, epidermal cell size and xyloglucan endotransglycosylase activity through the growing zone of ageing maize leaves. J Exp Bot 47(296): 339–347.

[34] Saghai-MaroofMA, SolimanKM, JorgensenRA, AllardRW (1984) Ribosomal DNA spacer-length polymorphisms in barley: Mendelian inheritance, chromoso- mal locations and population dynamics. Proc Natl Acad Sci U S A 81(24): 8014–8018.609687310.1073/pnas.81.24.8014PMC392284

[35] CloughSJ, BentAF (1998) Floral dip: a simplified method for agrobacterium-mediated transformation of *Arabidopsis thaliana* . Plant J 16(6): 735–743.1006907910.1046/j.1365-313x.1998.00343.x

[36] UlmasovT, HagenG, GuilfoyleTJ (1997) ARF1, a transcription factor that binds to auxin response elements. Science 276(5320): 1865–1868.918853310.1126/science.276.5320.1865

[37] UlmasovT, HagenG, GuilfoyleTJ (1999) Dimerization and DNA binding of auxin response factors. Plant J 19(3): 309–319.1047607810.1046/j.1365-313x.1999.00538.x

[38] UlmasovT, MurfettJ, HagenG, GuilfoyleTJ (1997) Aux/IAA proteins repress expression of reporter genes containing natural and highly active synthetic auxin response elements. Plant Cell 9(11): 1963–1971.940112110.1105/tpc.9.11.1963PMC157050

[39] GuilfoyleTJ, HagenG (2007) Auxin response factors. Curr Opin Plant Biol 10(5): 453–460.1790096910.1016/j.pbi.2007.08.014

[40] KrizekBA (1999) Ectopic expression of *AINTEGUMENTA* in *Arabidopsis* plants results in increased growth of floral organs. Dev Genet 25: 224–236.1052826310.1002/(SICI)1520-6408(1999)25:3<224::AID-DVG5>3.0.CO;2-Y

[41] MizukamiY, FischerRL (2000) Plant organ size control: *AINTEGUMENTA* regulates growth and cell numbers during organogenesis. Proc Natl Acad Sci U S A 97: 942–947.1063918410.1073/pnas.97.2.942PMC15435

[42] HoriguchiG, KimGT, TsukayaH (2005) The transcription factor *AtGRF5* and the transcription coactivator *AN3* regulate cell proliferation in leaf primordia of *Arabidopsis thaliana* . Plant J 43(1): 68–78.1596061710.1111/j.1365-313X.2005.02429.x

[43] KimJH, KendeH (2004) A transcriptional coactivator, *AtGIF1*, is involved in regulating leaf growth and morphology in *Arabidopsis* . Proc Natl Acad Sci U S A 101(36): 13374–13379.1532629810.1073/pnas.0405450101PMC516574

[44] ChoHT, CosgroveDJ (2000) Altered expression of expansin modulates leaf growth and pedicel abscission in *Arabidopsis thaliana* . Proc Natl Acad Sci U S A 97(17): 9783–9788.1093194910.1073/pnas.160276997PMC16942

[45] WangYJ, DengDX, ShiYT, MiaoN, BianYL, et al (2012) Diversification, phylogeny and evolution of *auxin response factor* (*ARF*) family: insights gained from analyzing maize *ARF* genes. Mol Biol Rep 39(3): 2401–2415.2166710710.1007/s11033-011-0991-z

[46] ShenCJ, WangSK, BaiYH, WuYR, ZhangSN, et al (2010) Functional analysis of the structural domain of ARF proteins in rice (*Oryza sativa* L.). J Exp Bot 61(14): 3971–3981.2069341210.1093/jxb/erq208PMC2935870

[47] WuJ, WangFY, ChengL, KongFL, PengZ, et al (2011) Identification, isolation and expression analysis of *auxin response factor* (*ARF*) genes in Solanum lycopersicum. Plant Cell Rep 30(11): 2059–2073.2173523310.1007/s00299-011-1113-z

[48] MunJH, YuHJ, ShinJY, OhM, HwangHJ, et al (2012) Auxin response factor gene family in Brassica rapa: genomic organization, divergence, expression, and evolution. Mol Genet Genomics 287(10): 765–784.2291530310.1007/s00438-012-0718-4PMC3459075

[49] HaCV, LeDT, NishiyamaR, WatanabeY, SuliemanS, et al (2013) The auxin response factor transcription factor family in soybean: genome-wide identification and expression analyses during development and water stress. DNA Res 20(5): 511–524.2381091410.1093/dnares/dst027PMC3789561

[50] MizukamiY (2001) A matter of size: Developmental control of organ size in plants. Curr. Opin. Plant Biol 4: 533–539.10.1016/s1369-5266(00)00212-011641070

[51] Niklas KJ (1994) Plant Allometry: The Scaling of Form and Process. Chicago: The University of Chicago Press.

[52] Esau K (1943) Ontogeny of the vascular bundle in *Zea mays*. Hilgardia 15, 327–368.

[53] EvertRF, RussinWA, BosabalidisAM (1996) Anatomical and ultrastructural changes associated with sink-to-source transition in developing maize leaves. Int J Plant Sci 157(3): 247–261.

[54] SharmanBC (1942) Developmental anatomy of the shoot of *Zea mays* L. Ann. Bot. (Lond.) 6(2): 245–284.

[55] SchnyderH, SeoS, RademacherIF, KuhbauchW (1990) Spatial distribution of growth rates and of epidermal cell lengths in the elongation zone during leaf development in Lolium perenne L. Planta. 181(3): 423–431.10.1007/BF0019589724196821

[56] MajeranW, FrisoG, PonnalaL, ConnollyB, HuangM, et al (2010) Structural and metabolic transitions of C4 leaf development and differentiation defined by microscopy and quantitative proteomics in maize. Plant Cell 22(11): 3509–3542.2108169510.1105/tpc.110.079764PMC3015116

[57] GuoM, SimmonsCR (2011) Cell number counts-The *fw2.2* and *CNR* genes and implications for controlling plant fruit and organ size. Plant Sci 181(1): 1–7.2160039110.1016/j.plantsci.2011.03.010

[58] GuoM, RupeMA, WeiJ, WinklerC, Goncalves-ButruilleM, et al (2013) Maize *ARGOS1 (ZAR1)* transgenic alleles increase hybrid maize yield. J Exp Bot doi:10.1093/jxb/ert370 10.1093/jxb/ert370PMC388329524218327

